# Effect of Li-ESWT on Testicular Tissue and Function in Androgen-Deficient Rat Model

**DOI:** 10.1155/2022/5213573

**Published:** 2022-03-14

**Authors:** Wen Jie Tian, Seung Hwan Jeon, Hyuk Jin Cho, U-Syn Ha, Sung-Hoo Hong, Ji Youl Lee, Jun Jie Piao, Zhong Cheng Xin, Ye Gang Chen, Hong Yu Feng, Sae Woong Kim, Woong Jin Bae, Mahadevan Raj Rajasekaran

**Affiliations:** ^1^Department of Urology, Second Hospital of Jilin University, China; ^2^Department of Urology, College of Medicine, The Catholic University of Korea, Seoul, Republic of Korea; ^3^Catholic Integrative Medicine Research Institute, The Catholic University of Korea, Seoul, Republic of Korea; ^4^China-Korea Joint Research Center for Male Reproductive and Sexual Medicine, Tianjin Institute of Urology, Tianjin, China; ^5^Department of Clinical Laboratory Science, Suwon Science College, Hwaseong, Republic of Korea; ^6^Department of Male Reproductive and Sexual Medline and Department of Urology, The Second Hospital of Tianjin Medical University, Tianjin, China; ^7^Department of Urology, San Diego School of Medicine, University of California, CA, USA

## Abstract

Low-intensity extracorporeal shockwave therapy (Li-ESWT), as a microenergy therapy, has the effects of inhibiting oxidative stress, antiapoptosis, and tissue repair, which is increasingly applied to a variety of diseases. Our research aims to explore the protective effects of Li-ESWT in the aging rat model and its possible molecular mechanism through in vivo and in vitro experiments. In vitro, TM3 Leydig cells incubated with H_2_O_2_ were treated with Li-ESWT at 4 energy levels (0.01, 0.05, 0.1, and 0.2 mJ/mm^2^). In vivo, we employed an androgen-deficient rat model to simulate male aging and treated it with Li-ESWT at three different energy levels (0.01, 0.05, and 0.2 mJ/mm^2^). Li-ESWT increased the expression of vascular endothelial growth factor (VEGF) in TM3 cells, improved antioxidant capacity, and reduced apoptosis, with the effect being most significant at 0.05 mJ/mm^2^ energy level. In androgen-deficient rat model, LI-ESWT can improve sperm count, motility, and serum testosterone level, enhancing tissue antioxidant capacity and antiapoptotic ability, and the effect is most significant at 0.05 mJ/mm^2^ energy level. Therefore, Li-ESWT at an appropriate energy level can improve sperm count, motility, and serum testosterone levels in androgen-deficient rat models, reduce oxidative stress in the testis, and increase antioxidant capacity and antiapoptotic abilities. The mechanism of this condition might be related to the increased VEGF expression in Leydig cells by Li-ESWT.

## 1. Introduction

Aging is a complex phenomenon attributed to developmental, genetic defects, environmental, disease, and hereditary factors, which accumulate adverse changes that increase disease risk [1]. Androgen-deficient is a common manifestation of aging in men, affecting up to 25% of older men, more than 10% of whom present as clinical symptoms of hypogonadism [2]. Johnson et al. [3] reported that the volume of testis increases in adolescence, peaks at the age of 30, and significantly declines after the age of 60. Testicular volume in elderly men is positively correlated with serum testosterone [4]. In previous studies, a comparative analysis [5] investigated the variation of testicular structure and function of 30 men age between 22-48 and 50-76 years, indicating that the average total number of Leydig cells in the oldest group decreased by 44% and thus affected the production of testosterone. However, some research results suggest the opposite conclusion [6, 7]. Although age-related regulation of the Leydig cell population remains controversial, some evidence in the literature shows that change in the maintenance of the redox balance within the Leydig cells affects their function. Previous research revealed that the superoxide content in aging Leydig cells is remarkably higher than in young Leydig cells [8]. Furthermore, the evidence of elevated levels of reactive oxygen species has been reported to be detected in 30-80% of infertile men's semen, showing that oxidative stress plays a critical role in male infertility. Oxidative stress can negatively affect fertility through a variety of pathways, interference with spermatozoa capacitation, and peroxidative damage to sperm membranes, proteins, and DNA, which are deleterious to the sperm's potential and decrease the chances of the fertilized egg developing into a healthy early embryo [9].

In urology, low-intensity extracorporeal shockwave therapy (Li-ESWT) is mainly used for Peyronie disease, chronic pelvic pain, and erectile dysfunction [10–12]. However, the effect of Li-ESWT on testicles and sperm is not well understood, so there are concerns about using Li-ESWT to treat male diseases. Studies have shown [13] that Li-ESWT has the effect of inhibiting oxidative stress and antiapoptosis. In our previous study, we found that Li-ESWT showed a dramatic promotion effect on the expression of vascular endothelial growth factor (VEGF) in the cavernous body [14, 15], and VEGF can stimulate the release of testosterone in Leydig cells [16]. Therefore, we hypothesized that Li-ESWT might positively affect testicles in older men.

The purpose of the present study was to investigate the restorative effects of Li-ESWT in the androgen-deficient rat model and to investigate the mechanism of Li-ESWT in TM3 Leydig cells in vitro.

## 2. Materials and Methods

### 2.1. In Vitro Immunofluorescence and Western Blot Testing Using TM3 Mouse Leydig Cells

TM3 cells, an immature mouse Leydig cell line (Korean Cell Line Bank, Seoul, Korea), were cultured in Dulbecco's modified Eagle's medium (DMEM)/F-12 medium (GIBCO, Life Technologies Co., USA) supplemented with 10% heat-inactivated fetal bovine serum (FBS; GIBCO) in a humidified atmosphere with 5% CO_2_/95% air at 37°C.

Cells (1 × 10^6^ cells) were plated on 6-well plates (Corning) in 10% FBS/DMEM/F-12 and subsequently incubated for 24 h. Oxidative cell stress was induced by treatment with 40 *μ*M H_2_O_2_ for 2 hours. Cells in each treatment group were given different energy levels of Li-ESWT (CENOWAVE; HNT MEDICAL Co., Ltd., Seoul, Korea) with 300 shocks each time, once a day, for a total of 7 times a week. TM3 cells were immobilized with 4% PFA for 15 min, then treated with cold methanol for 15 min, and permeated with 0.2% Triton X-100 in PBS at 4°C for 15 min. After washing with PBS, TM3 cells were incubated in a blocking solution (PBS containing 10% goat serum). TM3 cells were then combined with an anti-VEGF (1 : 500 dilution; Santa Cruz Biotechnology, USA) and *β*-actin (1 : 500 dilution; Santa Cruz Biotechnology, USA), staying overnight at 4°C. On the second day, TM3 cells were mixed with goat anti-rabbit IgG H&L (FITC) (1 : 100; Abcam, UK); after washing with PBS at room temperature for 2 h, the nuclei were identified by DAPI for 15 min and then rinsed with PBS and sealed.

Cells (1 × 10^6^ cells) were plated on 6-well plates (Corning) in 10% FBS/DMEM/F-12 and subsequently incubated for 24 h. Oxidative cell stress was induced by treatment with 40 *μ*M H_2_O_2_ for 2 hours. Cells in each treatment group were given different energy levels L with 300 shocks each time, once a day, for a total of 7 times a week. After processing, we gathered all cellular proteins by placing cells in a lysis buffer consisting of 0.1% sodium dodecyl sulfate in phosphate-buffered saline, followed by brief sonication. Protein concentration was identified by a bicinchoninic acid protein assay (Pierce Chemical Co., USA). Thirty micrograms of total cellular protein was separated by 12% SDS-polyacrylamide gel electrophoresis and then transferred to nitrocellulose membranes. Blots were probed with an antibody specific for the following proteins: *β*-actin (1:  1000 dilution; Santa Cruz Biotechnology, USA), HO-1 (1:  1000 dilution; Cell Signaling Technology, USA), Nrf2 (1:  500 dilution; Santa Cruz Biotechnology, USA), SOD (1 : 1000, dilution; Abcam, UK), NF-*κ*B (1 : 2000, dilution; Abcam, UK), and COX-2(1 : 1000 dilution; Cell Signaling Technology, USA). The binding antibody of each blot was evaluated by enhancing chemiluminescence (Western blot detection kit; Amersham Pharmacia Biotech, USA), which was assessed with horseradish peroxidase-conjugated secondary antibody.

### 2.2. Animal Groups and Treatment Protocol

This study was investigated in strict accordance with the recommendations in the Guide for the Care and Use of Laboratory Animals of the National Institutes of Health. The protocol was approved by the Institutional Animal Care and Use Committee in School of Medicine, The Catholic University of Korea (CUMC-2019-0072-03).

Male Sprague-Dawley (SD) rats 270-300 g (8 weeks of age) were randomly divided into four groups (6 rats in each group), which were submitted to (1) receive an intramuscular injection of normal saline (control); (2) receive a subcutaneous injection of an LHRH agonist (leuprolide acetate, Leuplin®; Takeda Pharmaceutical Co., Osaka, Japan) for four weeks to induce androgen-deficient (Leuplin); (3) after induction of androgen-deficient, 0.01 mJ/mm^2^ Li-ESWT was used for four weeks, once a week, 300 shocks each time (ESWT_0.01); (4) after induction of androgen-deficient, 0.05 mJ/mm^2^ Li-ESWT was used for 4 weeks with the same frequency (ESWT_0.05); and (5) after induction of androgen-deficient, 0.2 mJ/mm^2^ Li-ESWT was used for 4 weeks with the same frequency (ESWT_0.2). After 4 weeks, the animals in all groups were sacrificed, and the testes, epididymides, and blood samples were obtained.

### 2.3. Evaluation of Sperm Count and Motility in Caudal Epididymis

The right epididymis tissue was collected and minced and placed in normal saline containing 0.5% bovine serum albumin at 37°C and filtered. The sperm suspension was placed on preheated glass slides at 37°C. The sperm count was measured by Neubauer hemocytometer under 400x light microscope. The sperm count represented the number of sperm in 1 ml medium. Freshly collected left epididymis tissue was used for sperm motility analysis. Motile sperm percentage is more than 300 sperm randomly selected under the microscope, counting the motile sperm rate [17]. Each sample was counted three times.

### 2.4. Measurement of Germinal Cell Layer Thickness

Testicles were collected, washed with precooled PBS, and immediately impended in 4% paraformaldehyde for over 24 hours. The testicular tissue was corrected and placed into an automatic tissue processor for gradient ethanol dehydration. The sample was embedded in paraffin and cut into 4 *μ*m sections. Testicular specimens were dewaxed with xylene and ethanol, stained with hematoxylin and eosin, dehydrated, and fixed. Morphological changes of the testis were observed under a microscope, and the thickness of germinal cell layer was measured at 10 representative sites in the seminiferous tubules at random to complete image collection and analysis [18].

### 2.5. Serum Testosterone Levels

Before the rats were sacrificed, venous blood of inferior vena cava was taken, and serum testosterone level was measured by testosterone ELISA kit (Competitive ELISA, Immobilized antigen, RTC001R, BioVendor, Czech Republic). Place 10 *μ*l of sample (each specimen has three wells) with new disposable tips into appropriate wells dispensed in 100 *μ*l of incubation buffer into each well. Added was 50 *μ*l enzyme conjugate into each well which was incubated for 60 min at room temperature. This was discarded and well rinsed 4 times with diluted washing solution (300 *μ*l per well). Then, 200 *μ*l of substrate solution was added to each well and incubated standing for 30 min. The reaction was stopped by adding 50 *μ*l of stop solution to each well and the absorbance determined for each well at 450 nm. Repeat the test 3 times.

### 2.6. Measurement of Oxidative Stress

We used 8-hydroxy-2-deoxyguanosine (8-OHdG) level as a biomarker to detect DNA damage in testicular tissue and detected antioxidant levels in vivo by measuring superoxide dismutase (SOD) in testicular tissue. Total DNA was extracted from the testis using the DNeasy Blood & Tissue Kit (Qiagen, Valencia, CA, USA) and DNA oxidation Kit (Highly Sensitive 8-OHdG Check ELISA; Japan Institute for the Control of Aging, Fukuroi, Japan). After adding 3,3′,5,5′-tetramethylbenzidine for color development, the absorbance was measured at 450 nm. The tissue sample concentrations were measured using standard curves and DNA concentrations were corrected. The SOD activity (CuZnSOD and Mn SOD) in tissues was measured by SOD Assay Kit-WST (DG-SOD400, 400 tests, Dojindo), and the reduction rate of nitroblue tetrazolium mediated by superoxide was monitored by spectrophotometer at 450 nm.

### 2.7. TUNEL Staining

Apoptotic cells were detected in situ by indirect TUNEL assay using anti-digoxin antibody bound to fluorescein reporter molecule. Testicular tissue sections were blocked with 0.1% Triton X-100 for 5 minutes and then washed with PBS. Terminal deoxyribonucleotidyl transferase-mediated dUTP-digoxigenin nick-end labeling (TUNEL, ApopTag In Situ Apoptosis Detection Kits, Millipore, MA, USA) detection solution was dropped on each section and then incubated at 37°C in the dark which lasted for an hour. After rinsing with PBS, DAPI nuclei were stained for 5 minutes. After rinsing with PBS, sections were fixed with 50% glycerol. For the control group, the TUNEL solution was replaced by PBS. The sections were observed under a fluorescence microscope.

### 2.8. Animal Testicular Tissue Western Blot Analysis

We collected testicular histone proteins from each group, placed the crushed testicular tissue in a phosphate-buffered saline solution consisting of 0.1% sodium dodecyl sulfate, and then performed a brief ultrasound. The protein concentration was determined by the diphenylphenol acid protein assay (Pierce Chemical Co., USA). Thirty micrograms of total testicular tissue protein was separated by 12% SDS-polyacrylamide gel electrophoresis and transferred to nitrocellulose membranes. Specific antibodies were used to detect the following proteins: *β*-actin (1 : 1000 dilution; Santa Cruz Biotechnology, USA), HO-1 (1 : 1000 dilution; Cell Signaling Technology, USA), Nrf2 (1 : 500 diluted; Santa Cruz Biotechnology, USA), SOD (1 : 1000, dilution; Abcam, UK), BCL-xL (1 : 1000 dilution; Cell Signaling Technology, USA), Bax (1 : 1000 dilution; Cell Signaling Technology, USA), and Cleaved Caspase-3 (Caspase-3) (1 : 1000 dilution; Cell Signaling Technology, USA). The binding antibody of each blot was evaluated by enhancing chemiluminescence (Western blot detection kit; Amersham Pharmacia Biotech, USA), which was assessed with horseradish peroxidase-conjugated secondary antibody.

### 2.9. Statistical Analysis

Statistical analyses were carried out using SPSS 16.0 (SPSS Inc., Chicago, USA). The data was expressed as mean ± standard deviation. ANOVA test was used for data conforming to normal distribution, and the Scheffe test was used for comparison between groups. *P* < 0.05 was considered significant.

## 3. Results

### 3.1. Protective Effect of Li-ESWT on TM3 Leydig Cells in Vitro

Western blot analysis was conducted to determine whether Li-ESWT could prevent oxidative stress damage of TM3 Leydig cells induced by H_2_O_2_. As shown in Figure 1(a), compared with normal TM3 Leydig cells, the expression of Nrf2/HO-1 and SOD decreased significantly after incubation with H_2_O_2_ (*P* < 0.01). The expression level increased after Li-ESWT treatment, and the increase was most significant at 0.05 mJ/mm^2^ energy level (*P* < 0.01), which is also confirmed by quantitative analysis in Figure 1(b).

At the same time, as shown in Figure 1(c), NF-*κ*B/COX-2 expression was significantly increased after H_2_O_2_ incubation compared with normal TM3 Leydig cells (*P* < 0.01). This indicated increased apoptosis. The expression decreased after Li-ESWT treatment, and the decrease was most significant at 0.05 mJ/mm^2^ level (*P* < 0.01), which was also confirmed by the quantitative analysis in Figure 1(d). These results indicated that Li-ESWT could effectively prevent oxidative stress injury and reduce apoptosis of TM3 Leydig cells induced by H_2_O_2_, and the effect was most obvious at the energy level of 0.05 mJ/mm^2^.

### 3.2. Effect of Li-ESWT on VEGF Expression in TM3 Leydig Cells in Vitro

The effect of Li-ESWT on VEGF expression in TM3 Leydig cells was analyzed by immunofluorescence staining. As shown in Figure 2(a), compared with normal TM3 Leydig cells, the VEGF expression was significantly reduced after incubation with H_2_O_2_ (*P* < 0.01). The expression level increased after Li-ESWT treatment, and the increase was most significant at 0.05 mJ/mm^2^ energy level (*P* < 0.01). The quantitative analysis in Figure 2(b) also confirmed this, with an approximately 4-fold increase in the expression. This suggests that Li-ESWT can effectively increase the expression of VEGF in TM3 Leydig cells damaged by oxidative stress.

### 3.3. In Vivo, Li-ESWT Preserves Testicular Function and Improves Serum Testosterone Levels

There was no significant difference in body weight among the groups.  Table 1 lists the average weight of the testis for each group. After 8 weeks, the androgen-deficient group had significantly less testicular weight than the normal control group (*P* < 0.01). After Li-ESWT treatment, the testis weight was increased and the energy level was significantly increased at 0.05 mJ/mm^2^ (*P* < 0.01).

The testicular structure was normal, with mature vas deferens and complete spermatogenic sequence. But as shown in Figure 3, the density of spermatogenic cells decreased significantly in the androgen-deficient group compared with the normal control group (*P* < 0.01), and tissue degradation and even incomplete spermatogenic sequence could be seen in some vas deferens. Li-ESWT treatment improved with a significant increase in energy levels at 0.05 mJ/mm^2^ (*P* < 0.01) (Table 1).

Serum testosterone levels were significantly lower in the androgen-deficient group than in the normal control group (*P* < 0.01), and it was improved after Li-ESWT treatment, but the degree of improvement in each group was not statistically significant compared with the androgen-deficient group (Table 1).

### 3.4. In Vivo, Li-ESWT Reduced Oxidative Stress and Apoptosis

ELISA showed that the mean expression of 8-OHdG (Figure 4(a)) in the androgen-deficient group was significantly higher than that in the normal group, while the mean expression of SOD (Figure 4(b)) was significantly lower. Li-ESWT treatment reversed and was most obvious at 0.05 mJ/mm^2^ energy level (*P* < 0.01).

As shown in Figure 4(c), the expression of Nrf2/HO-1 and SOD in the androgen-deficient group was significantly decreased compared with the normal group (*P* < 0.01). Li-ESWT treatment reversed and was most obvious at 0.05 mJ/mm^2^ energy level (*P* < 0.01) (Figure 4(f)).

At the same time, as shown in Figure 4(e), the expression of Caspase-3 and Bax was significantly increased in the androgen-deficient group compared with the normal group, while the expression of Bcl-xL was significantly decreased, which was reversed after Li-ESWT treatment, and was most obvious at 0.05 mJ/mm^2^ energy level (*P* < 0.01) (Figure 4(f)).

Dark red apoptotic cells were observed in the testis during TUNEL assay (Figure 5(a)). The androgen-deficient group was significantly increased compared with the normal control group and decreased after Li-ESWT treatment, with a significant decrease in energy levels at 0.05 mJ/mm^2^ (*P* < 0.01), which is also confirmed by the quantitative analysis in Figure 5(b).

## 4. Discussion

In vitro cell experiments in this study, we set Li-ESWT at 4 energy levels (0.01, 0.05, 0.1, and 0.2 mJ/mm^2^). The results suggested that Li-ESWT could increase the expression of VEGF in TM3 cells, improve antioxidant capacity, and reduce apoptosis, and the effect was most significant at the energy level of 0.05 mJ/mm^2^. In androgen-deficient rat model, we set the Li-ESWT at 3 energy levels (0.01, 0.05, and 0.2 mJ/mm^2^). The results suggested that Li-ESWT could improve the sperm count, motility, serum testosterone level, tissue antioxidant capacity, and antiapoptotic ability. The effect was most significant at 0.05 mJ/mm^2^ energy level.

The transcription factor Nrf2 is a redox-sensitive transcription factor. It regulates the expression of HO-1 and confers cytoprotection against oxidative stress [19, 20]. Activation of Nrf2/HO-1 pathway can lead to increased SOD level in mouse kidneys [21, 22]. Previous research has shown that Nrf2 expression and related genes exhibit an age-dependent decrease in aged rats [23, 24]. This was consistent with our results. In androgen-deficient rat model, Nrf2/HO-1 expression and SOD level in rat testicular tissue were decreased, and the oxidative damage marker 8-OHdG was significantly increased, which was improved after Li-ESWT treatment. In our previous study [25], it was found that the expression level of Nrf2/HO-1 in TM3 stromal cells significantly decreased after oxidative stress. In the present research, the expression of Nrf2/HO-1 in TM3 cells was decreased after H_2_O_2_ treatment, while the expression level was increased after Li-ESWT treatment, which was consistent with the results of previous studies.

Apoptosis plays multiple roles in the normal growth and development of individual organisms and critical roles in maintaining normal, balanced homeostasis; however, excessive spontaneous apoptosis by generating increased intracellular reactive oxygen species production may cause organ dysfunction. Abbate et al. [26] have suggested that the expression of COX-2 in nonmyocytes in acute myocardial infarction was correlated with the induction of inflammation and severity of apoptosis. COX-2 expression is regulated by various transfactors, such as NF-*κ*B, which can bind to corresponding promoter regions to regulate transcription [27, 28]. COX-2 overexpression is associated with activation of NF-*κ*B signaling pathway [29]. In our cell experiments, NF-*κ*B and COX-2 were significantly increased after H_2_O_2_ treatment and decreased after Li-ESWT treatment. At the same time, the expression of TUNEL index, Caspase-3, and Bax was significantly increased, while the expression of Bcl-xL was significantly decreased in the androgen-deficient animal model. However, these changes can be reversed with Li-ESWT treatment, and the Bax/Bcl-xL ratio was reduced. Therefore, we believe that Li-ESWT can reduce tissue oxidative stress and apoptosis, improve antioxidant capacity and stromal cell activity, and at the same time increase serum testosterone level, further promoting sperm production.

Li-ESWT is an acoustic wave that produces mechanical forces to produce shear stress on the cell membrane, cytoskeleton, and extracellular matrix, thereby exerting biological effects [30, 31]. It has been reported that Li-ESWT can stimulate the upregulation of tissue repair markers such as VEGF [32–34] and reduce oxidative stress [35]. In our in vitro cell experiments, it was found that VEGF expression in TM3 cells decreased after H_2_O_2_ treatment and significantly increased after Li-ESWT treatment. Studies have shown that VEGF subtypes, as a gene regulator, are necessary for the maintenance of spermatogonia, sperm production, and male fertility [16]. Therefore, according to the results of this experiment, we believe that Li-ESWT may play an active role in testis by increasing the expression of VEGF in stromal cells. At the same time, we need to further study the mechanism.

Some studies have shown that Li-ESWT has a negative effect on testicles, contrary to our results [36–38], which may be related to the use of different energy levels. In our study, the optimal energy level obtained by cell and animal experiments was 0.05 mJ/mm^2^. In animal experiments, the results of 0.01 mJ/mm^2^ energy level were compared with the Leuplin group. Although the average value was changed, there was no statistical difference. Meanwhile, some results of 0.2 mJ/mm^2^ energy level were not statistically different from 0.05 mJ/mm^2^ energy level, but the average value was changed. This suggests that Li-ESWT energy level directly impacts its effect, and high energy level may reduce Li-ESWT effect. However, when Li-ESWT treated penis and other parts or even applied ESWT gravel energy to testis, the energy received by the testis was necessarily different from the energy given in our experiment, so the impact was unknown.

In this experiment, we intended to target aging male hypoandrogens with partial androgen deficiency rather than complete castration, so low-dose leuprorelin injection helped to establish this model. And we may study further experiments using older rat models. Although the average serum testosterone level increased after Li-ESWT treatment, there was no statistical difference. Meanwhile, we did not set sufficient energy level gradient in animal experiments. Although the results showed that the energy level of 0.05 mJ/mm^2^ was the best and different from other energy levels, this may not mean that this is the true optimal level, so we may need further research.

## 5. Conclusion

Both our experiments have confirmed that Li-ESWT with appropriate energy levels can improve sperm count, motility, and serum testosterone levels in androgen-deficient rat models. It can reduce oxidative stress in the testis and increase antioxidant capacity and antiapoptotic capacity, and the effect is most obvious at 0.05 mJ/mm^2^ energy level. We believe the mechanism underlying these findings may be related to the increase of VEGF expression in Leydig cells by Li-ESWT. Li-ESWT may serve as a new noninvasive and effective treatment to improve testicular function and sperm quality in middle-aged and elderly men. Meanwhile, we can also expect Li-ESWT to play a positive role in the oxidative stress lesions of the testis or other organs caused by obesity, metabolic diseases, or other injuries.

## Figures and Tables

**Figure 1:** Effect of Li-ESWT on protein expression in H_2_O_2_-treated TM3 Leydig cells in vitro. (a) The expression levels of Nrf2, HO-1, and SOD in cells of each group were detected by Western blot. (b) The expression of Nrf2, HO-1, and SOD in each group was quantitatively analyzed. (c) The expression levels of NF-*κ*B and COX-2 in each group were detected by Western blot. (d) The expression levels of NF-*κ*B and COX-2 in each group were quantitatively analyzed. ^∗^*P* < 0.01 compared with H_2_O_2_ group. ^#^*P* < 0.01 compared with ESWT_0.01, ESWT_0.1, and ESWT_0.2 group. ^&^*P* < 0.01 compared with ESWT_0.2. Normal control was normal TM3 Leydig cell group. H_2_O_2_ was the TM3 Leydig cell group treated with H_2_O_2_. ESWT_0.01 was the group of TM3 Leydig cells treated with H_2_O_2_ followed by 0.01 mJ/mm^2^ Li-ESWT treatment. ESWT_0.05, ESWT_0.1, and ESWT_0.2 were treated by the same method with different energy levels.

**Figure 2:** Effect of Li-ESWT on VEGF expression in H_2_O_2_-treated TM3 Leydig cells in vitro. (a) Representative images of VEGF expression in each group. Blue is DAPI, red is *β*-actin, and green is VEGF. (b) Positive rate of VEGF in each group. Each bar chart shows the mean (standard deviation). ^∗^*P* < 0.01 compared with H_2_O_2_ group. ^#^*P* < 0.01 compared with ESWT_0.01, ESWT_0.1, and ESWT_0.2 group. Normal control was normal TM3 Leydig cell group. H_2_O_2_ was the TM3 Leydig cell group treated with H_2_O_2_. ESWT_0.01 was the group of TM3 Leydig cells treated with H_2_O_2_ followed by 0.01 mJ/mm^2^ Li-ESWT treatment. ESWT_0.05, ESWT_0.1, and ESWT_0.2 were treated by the same method with different energy levels.

**Figure 3:** Pathological appearance of testicular tissue (hematoxylin and eosin staining). Compared with the normal control group, the germinal cell layer was narrower in the androgen deprivation group. The scale in the figure represents 100 *μ*m.

**Figure 4:** Comparison of 8-OHdG (a) and SOD (b) expression levels by ELISA. (c) The expression levels of Nrf2, HO-1, and SOD in each group were detected by Western blot. (d) The expressions of Nrf2, HO-1, and SOD in each group were quantitatively analyzed. (e) The expression levels of Bcl-xL, Bax, and Caspase-3 in each group were detected by Western blot. (f) The expressions of Bcl-xL, Bax, and Caspase-3 in each group were quantitatively analyzed. ^∗^*P* < 0.01 compared with the control group. ^#^*P* < 0.01 compared with Leuplin group. ^&^*P* < 0.01 compared with ESWT_0.01 and ESWT_0.2 groups.

**Figure 5:** TUNEL assay to detect the effect of Li-ESWT on apoptosis of testicular tissue. (a) The representative image of each group: blue is DAPI and red is TUNEL positive. (b) The positive rate of TUNEL detection in each group. ^∗^*P* < 0.01 compared with the control group. ^#^*P* < 0.01 compared with Leuplin group. ^&^*P* < 0.01 compared with ESWT_0.01 and ESWT_0.2 groups.

**Table 1:** Comparison of testicular health parameters. Data show mean ± standard deviation. Analysis of variance test. ^∗^*P* < 0.01 compared with the control group. ^#^*P* < 0.01 compared with Leuplin group.

	Testicular weight (g)	Sperm count (x10^6^/g cauda)	% of motile spermatozoa	Diameter of seminiferous tubules (*μ*m)	Serum testosterone (ng/ml)
Control	1.96 ± 0.09	233.3 ± 37.05	59.86 ± 11.31	301.58 ± 10.26	3.07 ± 0.33
Leuplin	1.14 ± 0.24^∗^	109.67 ± 31.34^∗^	21.88 ± 13.33^∗^	120.32 ± 12.55^∗^	1.28 ± 0.52^∗^
ESWT 0.01	1.25 ± 0.2	110 ± 16.09	25.45 ± 7.1	134.74 ± 8.33	1.30 ± 0.24
ESWT 0.05	1.50 ± 0.28^#^	161.1 ± 27.62^#^	39.13 ± 5.49^#^	178.36 ± 9.95^#^	1.67 ± 0.30
ESWT 0.2	1.46 ± 0.26	150.34 ± 30.86	33.03 ± 5.35	148.21 ± 12.21	1.58 ± 0.37

## Data Availability

The data used to support the finding of this study are available from the corresponding author upon request.
